This article has been retracted.

# Clinical Application of Artificial Intelligence: Auto-Discerning the Effectiveness of Lidocaine Concentration Levels in Osteosarcoma Femoral Tumor Segment Resection

**DOI:** 10.1155/2022/7069348

**Published:** 2022-03-28

**Authors:** Shuqin Ni, Xin Li, Xiuna Yi

**Affiliations:** ^1^Department of Anesthesiology, Yantaishan Hospital, Yantai 264003, Shandong, China; ^2^Department of Surgery, Jinyintan Hospital, Wuhan, Hubei 430022, China

## Abstract

Adolescents and children worldwide are threatened by osteosarcoma, a tumor that predominantly affects the long bone epiphysis. Osteosarcoma is the most common and highly malignant bone tumor in youngsters. Early tumor detection is the key to effective treatment of this disease. The discovery of biomarkers and the growing understanding of molecules and their complex interactions have improved the outcome of clinical trials in osteosarcoma. This article describes biomarkers of osteosarcoma with the aim of positively influencing the progress of clinical treatment of osteosarcoma. Femoral bone tumor is a typical condition of osteosarcoma. Due to the wide range of femoral stem types, complexities in the distal femur, and tumors in the rotor part of femur, physicians following the traditional clinical approach face difficulties in removing the lesion and fixing the femur with resection of the tumor segment. In this paper, the effect of small doses of different concentrations of lidocaine anesthesia in patients undergoing lumpectomy for osteosarcoma femoral tumor segments is investigated. A computer-based artificial intelligence method for automated determination of different concentration levels of lidocaine anesthesia and amputation of osteosarcoma femoral tumor segment is proposed. Statistical analysis is carried on the empirical data including intraoperative bleeding, intraoperative and postoperative pain scores, surgical operation time, postoperative complications, patient satisfaction, and local anesthetic dose. The results showed that the patients in the study group had low intraoperative bleeding, short operation time, low postoperative hematoma formation rate, high patient satisfaction, higher dosage of anesthetic solution, and low dosage of lidocaine. Results revealed that mean arterial pressure and heart rate in extubating and intubating were significantly lower in the observation group than in the control group, and a significant difference (*P* < 0.05) was observed between the two groups. This proves that the proposed algorithm can adequately reduce bleeding, alleviate postoperative pain, shorten operation time, reduce complications, accelerate recovery, and ensure better treatment results.

## 1. Introduction

Osteosarcoma is a disease of the bone first described in 1807 in the Boyle Lectures [1]. Osteosarcoma is the most common malignant bone tumor in this age group, with a higher incidence in males than in females. Osteosarcoma most often occurs in the long bone epiphysis (43% in the distal femur, 23% in the proximal tibia, and 10% in the proximal humerus). The main symptoms of osteosarcoma include swelling of the affected area, joint pain, and limitation of movement. Pathological examination provides definitive information on the diagnosis and tumor grading. Most osteosarcomas develop early pulmonary metastases. The five-year survival rate is higher in patients without metastases compared to those with pulmonary metastases. Neoadjuvant chemotherapy as well as surgical resection has increased the 5-year survival rate for such patients from 10% before 1970 to 50%–70%. microRNAs or miRNAs are highly conserved, endogenous, tightly regulated noncoding small RNAs (18–25 nucleotides) that target and inhibit mRNA transcription by direct degradation or inhibition of translation. Their expression is strictly regulated by epigenetics (e.g., DNA methylation, histone deacetylation, and other transcriptional regulatory mechanisms) [2–5]. miRNAs can inhibit the expression of oncogenes that play an important role in tumorigenesis. Taking osteosarcoma as an example, several studies have reported the expression profiles of different miRNAs in cell lines or samples. For example, miR-195, miR-99, miR-181, and miR-148a are upregulated in osteosarcoma, while others such as miR-539, miR-145, and miR-335 are downregulated in MG-63 human osteosarcoma cell line. As miRNA is a bone tumor marker, studies from the literature found that miR-195 levels in serum of osteosarcoma patients were lower than normal controls by real-time quantitative RT-PCR assay [6]. This indicates that miRNA has the potential to be used as a marker of osteosarcoma and can be used effectively for screening and monitoring of osteosarcoma. Serum miR-199a-5p was found at higher concentrations in osteosarcoma samples. miRNA (miR-21, miR-199a-3p, miR-143, miR-34, miR-140, and miR-132) expression levels were found to be higher in osteosarcoma patients, while miR-199a-3p and miR-143 in osteosarcoma patients had lower expression levels. Cytokines are small proteins secreted by monocytes and macrophages, among others, which are regulators of the host's response to trauma, infection, and immunity. Abnormally elevated plasma levels of proinflammatory cytokines have been associated with obesity, type 2 diabetes, atherosclerosis, rheumatoid arthritis, and cancer. Several studies have shown elevated levels of transforming growth factor (TGF-*β*) in patients with osteosarcoma compared to healthy controls. Osteosarcoma cells stimulate the production of protumor cytokines by mesenchymal stem cells (MSCs). The cells stimulate the production of IL-6 and vascular endothelial growth factor (VEGF) in MSCs through the medium of Saos-2 and U2 osteosarcoma cell lines. The stimulation effect can be neutralized by TGF-*β* antibodies. Drugs that inhibit TGF-*β* have also been used in preclinical studies and clinical trials. In contrast, VEGF has also been observed to be upregulated in several types of cancer, including osteosarcoma. The involvement of VEGF in angiogenesis has been used as a biomarker of prognosis in patients with osteosarcoma [7–9]. In addition, VEGF expression was also associated with overall disease-free survival, whereas patients with high VEGF expression had lower disease-free survival and overall survival, suggesting that VEGF may serve as a valid biomarker for osteosarcoma prognosis. Cytokine levels in osteosarcoma patients, including ILS-6, TGF-*β*, growth-related oncogenes, hepatocyte growth factor, chemokine ligand 16, end proteinase, matrix metalloproteinase-9, and platelet-derived growth factor-AA, were upregulated in the test group compared with normal controls. It was observed that enzyme-linked immunosorbent assay (ELISA) with MSC-based ILS-6, osteosarcoma proliferation, and metastasis was promoted. In [6] *β*-isomerized C-terminal peptide (*β*-CTx) and total type 1 procollagen aminoterminal peptide (tP1NP) were found to be significantly elevated by immunoassay of sera from osteosarcoma patients. Therefore, it is believed that these proteins could be used as osteosarcoma biomarkers. Abnormal TIM3 expression is associated with a variety of cancers, belongs to the family of molecules containing the immunoglobulin and mucin structural domains of T cells (TIM), and is expressed by a variety of immune cells including T cells, macrophages, dendritic cells, and natural killer cells. TIM3 is also expressed in human osteosarcoma cell lines. In addition, TIM3 has been found to be coexpressed with Slug, Snail, and Smad, which have been detected in osteosarcoma patients [10–12]. Therefore, TIM3 is expected to be used as a tool for the diagnosis and treatment of osteosarcoma. Matrix metalloproteinases (MMPs) belong to a family of zinc-dependent endopeptidases that are secreted by macrophages and neutrophils and are involved in a variety of physiological and pathological processes including extracellular matrix (ECM) degradation and remodeling, morphogenesis, wound healing, tissue repair, and remodeling. In addition, MMPs play a key role in tumor progression by activating cell growth, migration, invasion, metastasis, and angiogenesis. A study showed a significant correlation between MMP-9 expression and osteosarcoma risk in Asian and non-Asian populations [13].

Lidocaine is a local anesthetic with anesthetic and analgesic effects. Intravenous lidocaine can increase the risk of cardiac arrhythmias due to elevated blood concentrations. Transdermal topical administration, on the other hand, avoids hepatic first-pass effects, increases local drug concentrations at the site of pain, decreases systemic plasma concentrations of lidocaine, and reduces systemic adverse effects while also improving patient safety and compliance. Topical lidocaine formulations have been shown to exert analgesic effects by blocking voltage-gated sodium channels (Nav), effectively reducing abnormal peripheral nerve discharge, and decreasing peripheral sensitization. Lidocaine gel/ointment can be applied directly to the painful skin area, and in order to keep the gel in contact with the skin and enhance permeability, it is often used in combination with a closed dressing; however, the closed dressing is less tolerable due to the lack of breathability, easy to cause local burning sensation, and troublesome to use, so the lidocaine patch with a protective backing layer was created [14, 15]. The molecular formula of lidocaine is shown in Figure 1.

In March 1999, the U.S. Food and Drug Administration (FDA) approved lidocaine patch 5% for the treatment of postherpetic neuralgia (PHN). In Europe, the product was approved for marketing in the EU in 2007 under the name lidocaine patch 5%, and generic versions of lidocaine topical patches have been introduced into the market since then. In February 2018, the 1.8% lidocaine topical transdermal system was also approved by the FDA for PHN, and in the same year, lidocaine gel patches were marketed in China, filling a therapeutic gap in this area in China. The use of topical lidocaine patches (collectively, the above dosage forms) for the treatment of PHN has been supported by the consensus of clinical practice guidelines in China and abroad but has not been approved for other indications. Based on its effectiveness and safety in the treatment of PHN, lidocaine topical patches have also been widely used for other peripheral neuropathic pain conditions, such as diabetic peripheral neuropathic pain (DPNP) and postoperative or posttraumatic neuropathic pain, and even for localized injury-sensitive pain. However, the safety and efficacy in the treatment of other types of pain disorders are unclear, and there are few relevant studies in China.

The heterogeneity of osteosarcoma is a major factor in treatment outcome. Biomarkers can be used to diagnose patients with osteosarcoma, especially those with metastatic osteosarcoma, and biomarkers may be an effective way to diagnose osteosarcoma early and to identify potential therapeutic targets. Therefore, this paper reviews the research on biomarkers in cellular experiments, animal models, and histological specimens of osteosarcoma in this direction. Moreover, we study the dosage form characteristics, pharmacokinetics, safety, and efficacy of currently marketed lidocaine topical patches and their applications in the field of pain treatment, taking into account the latest advances, to provide a reference basis for its further in-depth research application. In this paper, a computer-based artificial intelligence method is proposed for the automated determination of different concentrations of lidocaine anesthesia in osteosarcoma femoral tumor segment resection, and the effectiveness of this method for determining different concentrations of lidocaine anesthesia applied in tumor resection surgery is demonstrated by experimental validation in relevant data.

The paper is organized into 4 sections.  Section 2 is about the literature review. The proposed method is discussed in Section 3. Experimentation and analysis are performed in Section 4 whereas conclusion is presented in the last section, Section 5.

## 2. Related Work

Pain has been listed as the “fifth vital sign” of the human body, yet the treatment of pain still faces great challenges in clinical practice. Among them, neuropathic pain is the common clinical pain caused by somatosensory system injury or disease. Chronic pain not only affects the patient's ability to sleep, work, and live, but also increases the incidence of depression, anxiety, and other emotional disorders, seriously affecting human health and quality of life. Therefore, early, adequate, and aggressive treatment of chronic neuropathic pain can effectively relieve pain and its accompanying symptoms, restore physical function, and improve quality of life. Although many drugs (e.g., anticonvulsants, antidepressants, and opioids) are available, systemic administration is often limited by adverse drug reactions, especially in elderly and frail groups. In contrast, topical administration has low systemic exposure and high safety [16], so topical dosage forms available for topical administration (e.g., gels, ointments, and patches) are receiving increasing attention from clinicians.

The femur is a favored site for bone tumors and tumor-like lesions in children, with diverse disease types, more homozygous lesions, and the site is deep, without obvious specific clinical symptoms, making differential diagnosis difficult. In children, benign lesions are common in the femur, including osteochondroma, osteoid osteoma, and osteoblastoma. The incidence is higher in males than females, and some literature reports that the most common benign bone tumor in children is osteochondroma, which accounts for 10% to 15% of bone tumors [6]. The incidence of benign tumors was higher in children with a wide variety of femoral tumors and tumor-like lesions, and the top three were osteoid osteoma, osteosarcoma, and osteochondroma, which were basically consistent with those reported in the literature [17–19]. Common signs of femoral tumors or tumor-like lesions in children include cystic expansion bone destruction, osteoblastoma, chondroblastoma, aneurysmal bone cyst, giant cell tumor of bone, bone cyst, and abnormal proliferation of bone fibers. Similarly, osteolytic bone destruction is a common sign of malignant bone tumors.

### 2.1. Tumor Segment of Femoral Bone

Common signs of bone destruction in children with femoral tumors or tumor-like lesions: cystic distensible bone destruction is the most common benign bone tumors and tumor-like lesions in children, including osteoblastoma, chondroblastoma, aneurysmal bone cyst, giant cell tumor of bone, bone cyst, and abnormal bone fiber proliferation disorder, while osteolytic bone destruction is a common sign of malignant bone tumors.  Figure 2 [20, 21] shows X-ray of right femoral neck osteoid osteoma of a male, 8 years old with cystic distensible bone destruction, all of which are benign bone tumors and tumor-like lesions with well-defined lesion extent.

Osteoblastic osteoma is most seen in adolescents under 25 years of age. The disease is more common in males and is more common in the lower extremities. Attack of the disease in childhood may lead to skeletal deformities. In children, endogenous chondrosarcoma and stromal ossification are rare, and the “fan-shaped sign” can be seen in their bone. Osteolytic destruction is a kind of malignant tumors; hence, osteosarcoma is characterized by osteolytic bone destruction with indistinct borders and worm-like or sieve-like destruction of the bone cortex, accompanied by tumor bone formation. When the lesion breaks through the articular surface, the continuity of the epiphyseal plate can be interrupted, and pathological fractures can sometimes occur in osteosarcoma that invades the epiphyseal plate and epiphysis. This increases the difficulty of diagnosis in children with osteosarcoma. In [22], image fusion technique based on advanced AI classifiers is proposed to diagnose osteosarcoma using the data of both CT and MRI images.

#### 2.1.1. Periosteal Reaction

When the outer periosteum of long bones is stimulated by a granulation tissue mass that breaks through the bone cortex, it can manifest as a periosteal reaction, such as laminar and onion skin-like. Malignant tumors, including osteosarcoma and lymphoma, can be seen with varying degrees of periosteal reaction, forming the Codman triangle. Typical eosinophilic granulomas in benign bone diseases may also show onionskin-like periosteal reaction with high density, no radiolucent bone pins, and well-defined margins. In case of eosinophilic granulomas, it is common that the extent of the bone destruction area exceeds limits and may be accompanied by a wide range of soft tissue masses or swelling, usually occurring in the epiphysis or bone ends of long bones. Malignant bone tumors have an incomplete periosteal response with radiolucent bone [23]. When the neoplastic periosteum is broken by the tumor, it can be deformed and disrupted, forming Codman's triangle, which can then be easily distinguished. In benign tumors and tumor-like lesions combined with pathological fractures, typically a thin periosteal reaction may appear.

#### 2.1.2. Intratumoral Calcification

When cartilage matrix calcium salt deposition or intratumoral tissue necrosis occurs, calcification signs may appear. Among benign tumors, chondroblastoma and osteoblastoma may show speckled calcification, which can be better visualized by high-resolution CT. Osteoblastoma and osteoblastoma can show speckled calcification in the nest. Among benign bone tumors, chondroblastoma is most often found in the epiphysis of long bones and can involve the epiphysis across the epiphyseal plate. Chondroblastoma can be differentiated from malignant bone tumors such as chondrosarcoma with incomplete circumferential calcification, low density, and indistinct margins.

#### 2.1.3. Fluid-Fluid Plane

Benign tumor-like lesions of aneurysmal bone cysts often show fluid-fluid plane. The principle is due to the separation of plasma and cells in the blood of the cyst and the formation of a partition interface after the bottom of cell precipitation. Aneurysmal bone cysts show typical fluid-fluid plane in CT and MRI, but fluid-fluid plane is not unique like that of aneurysmal bone cysts. The giant cell tumor of bone, osteoblast, and/or hemorrhage may cause this phenomenon.

#### 2.1.4. Focal Boundaries

Benign bone tumors and tumor-like lesions have clear boundaries due to slow development. The obvious sclerotic edges are often seen on X-ray and CT, while malignant tumors, such as osteosarcoma, chondroblastoma, and nonossifying fibroma, have clear sclerotic edges [24]. Osteochondroma is the most common benign bone tumor in children, preferably in boys, with the femur being the most common. Retrospective analysis of patients likewise revealed that osteochondroma is the most prevalent benign tumor. Osteochondroma occurs near the epiphysis of the long bones and presents as a bony redundancy with a cartilaginous cap and a well-defined lesion. The diagnosis of osteochondroma is established by X-ray plain film before surgery. Bone fibro dysplasia and aneurysmal bone cysts can be seen with clear sclerotic edges and internal segregation-like changes. CT and MRI are more advantageous in showing details of the lesion.

#### 2.1.5. Soft Tissue Changes

Benign bone tumors or tumor-like lesions may show soft tissue changes, including edema or mass formation, such as osteoid osteoma, chondroblastoma, and eosinophilic granuloma. Soft tissue swelling can be seen around osteoid osteoma and simple bone cysts combined with pathologic fractures, consistent with the literature. Typical childhood eosinophilic granuloma can be seen as soft tissue mass formation, but unlike malignant tumors, soft tissue masses have clear and smooth borders. The tissues are generally thin, elongated, and evenly encircle areas of bone destruction. Eosinophilic granuloma can be seen as an obvious elongated soft tissue mass that evenly encases the bone destruction area and can be seen as soft tissue swelling of varying degrees. Osteosarcoma is the most common malignant bone tumor of the long bones of the extremities in children, preferably in the epiphysis, and is characterized by osteolytic destruction and soft tissue masses within the verrucous bone. Osteosarcoma can be seen as soft tissue masses of varying sizes, with poorly defined borders and progressive enlargement [24].

### 2.2. Lidocaine Anesthesia

Local anesthetic lidocaine is a sodium channel blocker with membrane stabilizing effects and is used in antiventricular arrhythmias. In recent years, as pharmacological research and clinical applications continue to advance, lidocaine also has immune system regulatory functions and exerts anti-inflammatory effects in several parts of the inflammatory response. Its significant inhibitory effects on the inflammatory response, acute lung injury, sensitizing effects on anticancer drugs, bacterial inhibition, cerebral protection, and reduction of postoperative cognitive dysfunction (POCD) have received attention from clinical scholars and are reviewed below. Lidocaine has broad-spectrum antiarrhythmic effects. Ventricular arrhythmias include ventricular asystole, ventricular tachycardia, ventricular flutter, and ventricular fibrillation. The latter three characteristics are known as malignant arrhythmias and are an independent risk factor for sudden cardiac death, and malignant ventricular arrhythmias often lead to hemodynamic deterioration, accelerated progression, and even life-threatening conditions. Lidocaine is a class IB antiarrhythmic drug, which selectively acts on Purkinje fibroblasts and ventricular myocytes, slowing down the rate of 4-phase depolarization, reducing the autoregulation of Purkinje fibroblasts, promoting K+ efflux, shortening the action potential time course, and relatively prolonging the effective induction period. It is often used in the prevention and treatment of ventricular arrhythmias. Lidocaine slows cardiac conduction, inhibits cardiac contractility, and decreases cardiac output. Lidocaine has been used for a long time and has more experience in clinical antiarrhythmic use. In the face of ventricular arrhythmias, clinicians often choose lidocaine to control them, and its effectiveness and safety are high. Lidocaine can prevent excessive inflammatory responses. Many studies have shown that lidocaine is very effective in preventing and combating trauma or endotoxin-induced inflammatory responses [25]. Lidocaine is a membrane stabilizer that inhibits neutrophil (PMN) adhesion and aggregation, reduces oxygen radical and protein hydrolase release, stabilizes cell membranes, regulates cytokines, and suppresses excessive inflammatory responses. Inflammatory mediators LB4 and interleukin 1*α* (IL-1*α*) are strong PMN chemotactic agents, inducing PMN edge, degranulation, exudation, superoxide production, and increasing vascular permeability in concert with prostaglandin E2 [24, 26]. In vitro incubation of monocytes with different concentrations (2–20 mol/L) of lidocaine significantly inhibited the release of LB4 and IL-1*α*, and micromolar concentration levels of lidocaine inhibited the release of histamine from leukocytes, mast cells, and basophils, suggesting that lidocaine can inhibit the release of some key inflammatory mediators and exert anti-inflammatory effects. In clinical applications, several studies have found that intraoperative intravenous infusion of lidocaine can modulate patients' immune function and accelerate their postoperative recovery. Intraoperative lidocaine infusion in patients undergoing colorectal surgery was found to accelerate the recovery of enhanced gastrointestinal function and significantly shorten the length of hospital stay, while intravenous lidocaine infusion significantly reduced the expression levels of IL-6 and IL-8, complementing C3a, CD-11b, etc. in plasma. In [27], it is reported that in a prospective randomized double-blind controlled trial, intravenous lidocaine infusion was given to outpatient laparoscopic patients, and it was found that the postoperative recovery index was significantly higher in the lidocaine group. Besides, it was observed that intravenous lidocaine infusion significantly reduced the length of hospital stay and reduced the dose of opioids used by the patients. There are complications that prevent the occurrence of phlebitis during Patient-Controlled Intravenous Analgesia (PCIA) while adding lidocaine to the intravenous analgesic pump. It may be due to the action of lidocaine on vascular endothelial cells and peripheral nerve receptors near the venipuncture site, which dilates the blood vessels and inhibits the irritation response of the vein wall to the cannula needle and the release of inflammatory factors from vascular endothelial cells. The dilated blood vessels accelerate blood flow and make platelets less likely to aggregate, thus preventing the formation of microthrombi and the occurrence of phlebitis. Chemotherapy-induced phlebitis often occurs in clinical practice, and some studies have shown that the use of low-dose lidocaine plus dexamethasone in the perioperative period to prevent chemotherapeutic phlebitis has significant efficacy [28]. In conclusion, perioperative low-dose intravenous lidocaine can reduce the inflammatory response due to surgery, reduce the amount of anesthesia and analgesics used during surgery, and relieve postoperative pain. Lidocaine, a commonly used amide local anesthetic, has been shown to have anti-inflammatory effects, and perioperative intravenous infusion of lidocaine can reduce postoperative pain, decrease the use of opioid analgesics, reduce the inflammatory response of the body, accelerate the recovery of gastrointestinal function, and shorten the hospital stay of patients. Further study on the protective effect and mechanism of lidocaine on the decrease of immune function caused by surgical trauma can provide a new theoretical basis for the application of lidocaine in clinical anti-inflammatory treatment.

### 2.3. Artificial Intelligence Healthcare

Deep learning models can be flexibly scaled to huge data resources and improved by distributed dedicated hardware resources. The migration strategies can be introduced to easily improve the performance on more types and domains of data. Deep learning models have gradually replaced the traditional machine learning methods to effectively implement and utilize AI technology in healthcare. On the other hand, deep learning models have the flexibility to encode heterogeneous data, catering to the heterogeneous nature of medical data. In [24], a deep learning algorithm is trained using more than 17,000 facial images of patients to identify rare genetic syndromes with high accuracy. The research is based on the idea that various genetic syndromes exhibit unique facial features that can help clinicians make a diagnosis. Google Inc. released a model based on a deep learning approach that uses current and historical CT images of patients to predict lung cancer risk [29]. The block diagram of the intelligent medical system is shown in Figure 3. The model has been shown to achieve the best current results on 6,716 cases, outperforming human radiologists' diagnoses, especially in cases where historical CT image data are not available. The model provides an overall prediction of lung cancer malignancy and identifies less visible malignant tissue in the lung. The model also effectively incorporates historical scans to help predict lung cancer risk, given that historical data on the growth rate of malignant tissue in the lung can help predict malignancy.

DeepMind has released a new circulating neural network-based artificial intelligence algorithm [30] that can predict acute kidney injury lesions 48 hours before they occur. By incorporating AI algorithms and intelligent medical assistants, the system proposes a shift from a reactive to a preventive model of care. The AI-based model proposed in [26] can help improve patient care and reduce healthcare spending. Researchers at the Massachusetts Institute of Technology have developed a system to predict the characteristics of vocal cord disease [31]. Built on a dataset of more than 100 medical subjects, the system uses features automatically extracted from this data and then trained with high precision to classify patients with and without vocal cord nodules. The study takes full advantage of the data from the rise of wearable devices, with approximately one week of voice monitoring data and billions of samples for each subject in the dataset. The corresponding signals captured from small accelerometers and sensors mounted on the subject's neck overcome many of the drawbacks of traditional feature engineering methods for mining disease-causing features. The research aims to improve medical decision-making by replacing some of the steps with excessive manual input through the application of artificial intelligence in medicine. The greatest achievement of deep learning for image analysis is reflected in the field of computer vision research. Accordingly, medical image analysis technology has become the brightest calling card of artificial intelligence technology in the current medical field. The related technology excels in processing convolutional neural network models with spatially invariant data. Relying on image video analysis and parsing technology, it handles tasks such as target classification, target detection, and target segmentation, which are very effective in determining whether a patient's CT image contains malignant tumors and other diseases. Such computer vision-based image classification and target detection applications are useful in complex diagnoses in dermatology, radiology, and pathology as well [32]. For instance, in [33] a fully automated tool is proposed to assess viable and necrotic tumor in osteosarcoma, by utilizing 40 digitalized slide images and 13 machine learning models. Apart from the above-mentioned clinical decision-making systems, a large number of artificial intelligence-based clinical and healthcare systems have been proposed and simulated in clinical and wellbeing setups for cancer [34], diabetes mellitus [35], and wellness recommendations [36, 37].

## 3. Method

At present, the depth of anesthesia is monitored in a subjective way by observing the patient's signs that are more affected by drugs, surgical stimulation, and primary diseases, such as respiration, circulation, eyes, skin, digestive tract, and skeletal muscle tone. It can also be monitored in an objective way with the help of monitors, certain vital signs of the patient, etc., and a quantitative evaluation index is given. With this research work, an objective method is proposed utilizing AI classifiers on EEG data to accurately predict the depth of anesthesia. The approach is feasible to understand the current state of anesthesia of the patient and requires no advanced skill or professionalism. Detail of the model is presented in the following subsections.

### 3.1. Model Architecture

The method proposed in this paper is based on EEG signals and neural networks, which has the advantage of reflecting conscious activity and noninvasive characteristics and is one of the most promising methods in detecting the depth of anesthesia at present. The method architecture is shown in Figure 4.

### 3.2. Data Preprocessing

In places such as operating rooms, electroencephalogram (EEG) signals are susceptible to pulse interference caused by equipment such as high-frequency electric knives. The EEG signal is a low frequency signal, and the signal frequency band is generally 0.5∼35.0 Hz. According to the characteristics of EEG signal, the high frequency noise signal can be filtered out. For doing so, a corresponding low-pass filter is designed to retain the effective EEG signal. In the proposed method, the adaptive thresholding method is used to better overcome the pulse interference. The threshold is continuously adjusted to accommodate the whole signal change. The adaptive thresholding method first segments the EEG signal with each segment containing 0.5 s of data. The variance of one segment of data is multiplied by the scale factor and is used as a threshold value for the next segment of data. If the computed variance of the next segment of data is less than the threshold value, the data is modified and the threshold value is updated; otherwise, the segment of data is deleted. A 4^th^ order 47 Hz Butterworth low-pass filter is used to filter out the high frequency interference signal based on retaining the low frequency effective signal of EEG signal. As the EEG signals acquisition process is susceptible to the interference of 50 Hz industrial frequency signal, a 4^th^ order 50 Hz trap is used to filter out the interference of the industrial frequency signal. During the EEG signal acquisition process, it is also susceptible to interference from human movement, which generates baseline drift. The baseline drift will cause the EEG signal to drift up and down. However, the interference generated by human movement can be effectively removed by designing a high-pass filter with a 2^nd^ order 0.5 Hz Butterworth filter. The EEG signal processing flow is shown in Figure 5.

Periodogram spectrum estimation, when the signal sequence is of finite length, is given as

(1) $$\begin{array}{c} \hat{P}\left(w\right)=\frac{1}{N}{\left|\sum_{n=1}^{N}x\left(n\right){\text{e}}^{-jwn}\right|}^{2}. \end{array}$$

The periodogram method has low frequency resolution and simple calculation because of the power spectrum estimation. Given the poor spectral performance of the periodogram method, the variance characteristics of the periodogram are improved using the averaging method. To obtain the weighted overlapping averaging, the Welch averaging periodogram method is used. For *L* independent random variables *X*_1_, *X*_2_⋯*X*_*L*_ with same mean *μ* and variance *δ*^2^, the new random variable *X*=(*X*_1_+*X*_2_+⋯+*X*_*L*_)/*L* has mean *μ* and variance reduced by a factor of *L*. With the Welch averaging method segments *x*_*N*_*(n)*, the data in each segment overlap by *M* points for the number of segments *L* given as

(2) $$\begin{array}{c} L=\text{floor}\left(\frac{N-\text{lap}}{M-\text{lap}}\right), \end{array}$$

where lap is the number of overlapping data points to add a window *w*(*n*) to each segment of data and adding a Hanning window to improve the spectral distortion occurred due to a large side flaps of the rectangular window. The power spectrum is computed as

(3) $$\begin{array}{c} {\hat{P}}_{\text{PER}}^{i}\left(k\right)=\frac{1}{MU}{\left|\sum_{n=1}^{M-1}X_{N}^{i}\left(n\right)w\left(n\right)W_{M}{}^{-kn}\right|}^{2}. \end{array}$$

Thus, the average power spectrum obtained by the Welch averaging method is given as

(4) $$\begin{array}{c} {\hat{P}}_{PER\;}\left(k\right)=\frac{1}{MUL}\overset{L}{\underset{i=1}{\sum }}{\left|\sum_{n=1}^{M-1}X_{N}^{i}\left(n\right)w\left(n\right)W_{M}^{-kn}\right|}^{2}. \end{array}$$

The Welch averaging method has the characteristics of data overlapping and increasing number of segments and is, therefore, more computationally intensive. Let *P(k)* be the power spectrum of the Fourier transform of *N* points, and the formula to find the total power of the waveform from 0 to 30 Hz is given as

(5) $$\begin{array}{c} \text{Total}\_\text{Power}=\sum_{k=1}^{30\times N/s}P\left(k\right). \end{array}$$

### 3.3. Neural Networks

The back propagation (BP) neural network consists of an input layer, an implicit layer, and an output layer. The forward propagation of the working signal and the backward propagation of the error signal are continuously cycled to make the output of the network closer to the expectation until the error between the output of the network and the expected output is small enough or the iteration steps reach the preset limit. The construction of the BP network structure mainly includes the determination of the number of layers and hidden layer nodes of the BP network and the design of the input and output nodes. Through the determination of the number of hidden layers of BP, Hecht Nielsen proved that when each node has different thresholds, a continuous function in the closed region can be approximated by a network with one hidden layer [38]. Therefore, a three-layer BP neural network can accomplish any n-dimensional to m-dimensional mapping.

If the number of nodes in the hidden layer is too small, the training effect is poor and the training accuracy is not achieved, which reduces the prediction ability of the network, i.e., “underfitting”. Too many nodes in the hidden layer will lead to “overfitting”. In order to find a suitable number of nodes in the hidden layer, a smaller number of nodes in the hidden layer are used to train the network first. In case sufficient accuracy is not achieved, the number of nodes in the hidden layer is gradually increased, and then the network is retrained. Different numbers of hidden layer nodes have little effect on the generalization ability of the network. In the proposed method, the three-layered network is followed because of two main reasons: (1) in order to improve the generalization ability of the network, the training process uses validation method to check the generalization ability. After setting the max-failure times, if the parameter values during validation cause a continuous rise in the prediction error, the training is stopped. (2) A simpler anesthesia depth exponential function is used, which can be fitted by a three-layer BP network using a smaller number of nodes. Therefore, to reduce the network structure, a smaller network is used and the number of nodes in the hidden layer is set to 5.

The number of input and output nodes of the BP network is selected such that the number of input nodes depends on the dimensionality of the data source and the input feature vector. The anesthesia depth index is fitted by 3 parameters, spectral edge frequency (SEF), BETA-RATIO, and burst-suppression ratio (BSR); thus, the number of network input nodes is set to 3. The output of the network has only one parameter, i.e., the anesthesia depth evaluation value, which is a dimensionless value from 0 to 100, so the number of nodes in the output layer of the network is set to 1.

One of the considerations of this paper is to find out whether different excitation functions influence the generalization ability of the network or not; key focus is paid on the selection of the network excitation function. Since the bispectral index (BIS) function is a linear function, the final choice in this paper is the linear excitation function, PURELINE. The activation function is expressed as

(6) $$\begin{array}{c} y=f\left(\sum_{i=1}^{r}w_{i}x_{i}\right). \end{array}$$

The effect of different learning functions on the generalization ability of the network was examined. It was observed that training algorithms of the BP neural networks have a great impact on the generalization ability, convergence rate, and stability of the network. As it is difficult to predict how much time a training method consumed in training, the correlation coefficient of BIS was computed to select a suitable training function. Different training functions have different values of the correlation coefficient *r* between the fitted BIS and nonfitting BIS values. If the *r* values obtained for each validation sample of a certain training function are, as a whole, larger than the *r* values obtained for other training functions, it is assumed that the training function has a strong generalization ability. Although the algorithm with variable learning rate converges slowly, in some specific cases, the algorithm converges too fast. In such case, the training ends earlier and the obtained results do not reach the required target, thus missing the point that minimizes the error. Therefore, as a result it was decided to use the momentum BP algorithm trained with variable learning rate, which is one of the most commonly used training algorithms in BP networks.

## 4. Experimentation and Evaluation

The proposed method is evaluated by real data obtained from the patients suffering from osteosarcoma in the Yantaishan Hospital, Zhifu District, China. Details of the experiment and evaluation are presented in the following subsections.

### 4.1. Dataset

One hundred and five patients undergoing osteosarcoma femoral tumor segment amputation from January 2020 to January 2021 in Yantaishan Hospital were randomly divided into an observation group (58 patients) and a control group (57 patients). Inclusion criteria: both groups were patients undergoing osteosarcoma femoral tumor segment resection; patients were willing to cooperate with the study; patients had good communication skills; and patients were assessed as grade I to III by the American Society of Anesthesiologists. Exclusion criteria: patients with mental disorders; patients <18 years of age; patients with other serious diseases; patients with long-term sedation; patients with an operation time longer than 3 h; and patients with intraoperative accidents. The general data of the two groups were not significantly different (*P* > 0.05) and were comparable.

### 4.2. Experimental Setup

This experiment uses a hardware platform to collect dental data from the patient's mouth. First, the tongue depressor with camera is inserted into the patient's oral cavity, the high brightness LED is used for both the groups, the multifunctional monitor was connected after admission to the operating room, and intravenous inhalation anesthesia was given by tracheal intubation. In both groups, no sedative drugs were used before induction of anesthesia, and intravenous midazolam (dose 0.04 mg/kg), sufentanil (dose 0.4 *μ*g/kg), etomidate (dose 0.2 mg/kg), and cis-atracurium (dose 0.2 mg/kg) were given to patients for induction of anesthesia. After the disappearance of the lash reflex and general relaxation of patients, tracheal intubation was given, and the ventilator was connected. Anesthesia was maintained, using lidocaine every hour as per the proposed AI algorithm to automatically calculate the use of intermittent additional. Intraoperative additional lidocaine was used to maintain the EEG bispectrality index (BIS) at 40–55; the infusion of lidocaine was stopped 10 min before the end of surgery, and the infusion of sufentanil was stopped after the completion of skin sealing. At the end of surgery, when the patient's BIS was ≥80, he was resuscitated in the anesthesia resuscitation room. In the observation group, dexmedetomidine hydrochloride was given by intravenous pump at a dose of 0.5 *μ*g/kg for 15 min before the end of surgery. The control group was given an equal amount of saline in the same way. SPSS 20.0 software was applied for data analysis, and the measurement data were expressed as mean ± standard deviation. The *t*-test was used for comparison between the groups and the count data were expressed as number of cases (in %). The *χ*^2^ test was used for comparison where a value of *P* < 0.05 was considered significantly different.

### 4.3. Evaluation Metrics

The mean arterial pressure (MAP) and heart rate (HR) at different time points: the time of anesthesia, recovery time of spontaneous respiration, extubating time, and awakening time; the occurrence of agitation; and the incidence of complications in the two groups were used as observation indexes. Patients' agitation was evaluated by the following methods: patients who were able to cooperate quietly were evaluated as grade 0, patients who moaned intermittently were evaluated as grade 1, patients who moaned continuously were evaluated as grade 2, and patients who shouted and struggled were evaluated as grade 3 and were evaluated as severe agitation. Complications included hypoxemia, chills, hypotension, and choking cough.

### 4.4. Experimental Results

The MAP and HR of the two groups at different time points were compared before extubating at the end of surgery (T1). There was no significant difference between MAP and HR of the observation group and the control group (*P* > 0.05). However, MAP and HR of the observation group were significantly lower than those of the control group at the time of extubating (T2) and 5 min after extubating (T3) (*P* < 0.05); see Table 1.

Comparison of anesthesia-related indexes between the two groups: there was no significant difference in the anesthesia time, recovery time of spontaneous breathing, and extubating time in the observation group compared with the control group (*P* > 0.05), but the awakening time in the observation group was significantly shorter than that in the control group (*P* < 0.05); see Table 2.

The incidence of agitation in the observation group (60.3%) was significantly lower than that in the control group (82.5%) (*P* < 0.05); see Table 3.

There was no significant difference in the incidence of complications in the observation group (20.7%) compared with that in the control group (19.3%) (*P* > 0.05); see Table 4.

## 5. Conclusion

In the limb-preserving surgical treatment of femoral bone tumor, complete resection of the tumor segment, local bone graft, allograft or reimplantation after inactivation of the tumor segment, and fixation of the femur with appropriate internal fixation are required to restore lower limb function. In this study, patients with osteosarcoma femoral tumor segment amputation in Yantaishan Hospital were treated with lidocaine definite injection, and the results showed that MAP and HR in T2 and T3 were significantly lower in the observation group than in the control group, suggesting that lidocaine definite injection contributes to the hemodynamic stability of patients after general anesthesia. The analgesic effect may promote the stabilization of theophylline and aldosterone in patients' bodies after surgery and reduce the effect on patients' cardiovascular system. The awakening time of the observation group was significantly shorter than that of the control group, suggesting that the lidocaine definitive injection promoted the awakening of the patients, and its analgesic and sedative effects may have played an important role in the awakening of the patients. The incidence of agitation in the observation group was significantly lower than that in the control group, which further showed that lidocaine definitive injection helped to reduce the incidence of agitation in patients. This result has some differences with other types of postoperative patients under general anesthesia in the data, but the ability of lidocaine definitive injection to reduce the incidence of agitation in patients is consistent. The reason may be related to the type of surgery selected in this study and the selection of cases. The incidence of complications in the observation group was the same as that in the control group, suggesting that lidocaine definitive injection promotes patients' awakening through analgesia and sedation and reduces the incidence of agitation in patients, but has no significant side effects on patients, which is of great value in the clinical application for patients under general anesthesia. To summarize, the AI algorithm based on the automated determination of different concentrations of lidocaine dine injection applied to patients with osteosarcoma femoral tumor segment amputation proposed in this paper can help maintain the stability of MAP and HR of patients, reduce the incidence of agitation of patients, and have no significant side effects on patients. The method is significant for further promotion and application.

## Figures and Tables

**Figure 1:** Lidocaine molecular formula.

**Figure 2:** Male, 8 years old, X-ray of osteoid osteoma of the right femoral neck.

**Figure 3:** Intelligent medical system.

**Figure 4:** Model structure.

**Figure 5:** EEG signal preprocessing flow chart.

**Table 1:** Comparison of mean arterial pressure (MAP) and heart rate (HR) between the two groups at different time points (*x* ± *s*).

Group	Number of cases	MAP/mmHg			HR/(times/min-1)		
		T1	T2	T3	T1	T2	T3
Observation group	58	80.2 ± 11	81.6 ± 12.4	81.3 ± 12.1	80.7 ± 12.4	79.3 ± 12.9	82.2 ± 14.1
Control group	57	80.2 ± 11	109.8 ± 13.4	100.3 ± 12.7	81.2 ± 12.6	90.1 ± 13.5	93.6 ± 14.2

*t*		0.824	7.236	5.043	0.721	5.526	6.137
*P*		0.217	0.000	0.002	0.342	0.003	0.001

**Table 2:** Comparison of anesthesia-related indicators between the two groups [(*x* ± *s*), min].

Group	Number of cases	Duration of anesthesia	Recovery time of spontaneous breathing	Time to extubation	Time to awaken
Observation group	58	138.3 ± 15.5	11.3 ± 2.2	8.4 ± 2.3	19.2 ± 4.9
Control group	57	139.6 ± 16.8	11.2 ± 2.4	8.5 ± 2.6	35.4 ± 6.1

*t*		0.915	1.118	0.853	10.024
*P*		0.162	0.132	0.225	0.000

**Table 3:** Comparison of the occurrence of agitation during the awakening period between the two groups (cases, %).

Group	Number of cases	Level 0	Grade 1	Level 2	Grade 3	Total
Observation group	58	23 (39.7)	24 (41.4)	8 (13.8)	3 (5.2)	35 (60.3)
Control group	57	10 (17.5)	23 (40.3)	16 (28.1)	8 (14.0)	47 (82.5)

*t*						6.869
*P*						0.009

**Table 4:** Comparison of the occurrence of complications between the two groups (cases, %).

Group	Number of cases	Chills	Hypoxemia	Hypotension	Choking cough	Total
Observation group	58	2 (3.4)	4 (6.9)	3 (5.2)	3 (5.2)	12 (20.7)
Control group	57	3 (5.3)	3 (5.3)	2 (3.5)	3 (5.3)	11 (19.3)

*t*						0.035
*P*						0.852

## Data Availability

The datasets used during the current study are available from the corresponding author on reasonable request.
